The article "Temperature resistant anti-reflective coating on Si-wafer for long-wave infra-red imaging" was published in 2023. Journal: Heliyon.

# Temperature resistant anti-reflective coating on Si-wafer for long-wave infra-red imaging

**DOI:** 10.1016/j.heliyon.2023.e15888

**Published:** 2023-04-27

**Authors:** Phillip H. Papatzacos, M. Nadeem Akram, Olivier Hector, Frédéric Lemarquis, Antonin Moreau, Julien Lumeau, Per Ohlckers

**Affiliations:** a Department of MicroSystems, University of South-Eastern Norway, Borre, Norway; b Aix Marseille Univ, CNRS, Centrale Marseille, Institut Fresnel, Marseille, France

**Keywords:** Long wave IR, Anti-reflective coatings, Thermal camera, Microbolometers, Electron beam deposition, Si

## Abstract

A micromachined Silicon lid, sealed by CuSn solid liquid interdiffusion bonding is a promising approach for hermetic sealing of microbolometers for use in low-cost thermal cameras. However, since ∼30% of long-wave infrared light is reflected at an uncoated single Si-air interface, anti-reflective treatments are required. Traditional anti-reflective coatings are inapplicable since CuSn solid liquid interdiffusion bonding requires heating to about 270 °C and these multi-layer coatings fail due to differing coefficients of thermal expansion for the different layers and the substrate. For this purpose, an anti-reflective coating that maintains its anti-reflective properties after being heat-cycled to 300 °C has been developed. This coating was developed using a simple 2-layer structure composed of ZnS and YF_3_ and deposited at 100 °C. The development process that led to the successful coating has also been described in this paper. The final sample shows a 30% average increase in transmission in the 8–12 μm wavelength range as compared to an uncoated wafer.

## 1 Introduction

Infrared (IR) microbolometers have been developed which, when placed in an array, result in a thermal camera with low cost and no need for active cooling. These MicroBolometer Arrays (MBAs) therefore have the potential to bring thermal cameras to new application avenues, such as thermography for quality assurance and control, automated driver assistance systems in cars and unmanned aerial aircraft systems, as well as other surveillance, security, and safety applications [1].

Packaging of these MBAs, like most Micro-Electro-Mechanical Systems (MEMS), is challenging because these devices are sensitive and have strict requirements when it comes to processing techniques, processing temperature, and vacuum operating level [1]. One promising approach for encapsulating these MBAs is to use thin micromachined silicon as a cap and seal the package using CuSn Solid Liquid Interdiffusion bonding (SLID) (see Fig. 1). Silicon is chosen due to its relatively high transparency in the Long Wave InfraRed (LWIR) region and its long history of wide implementation in large-scale production [1]. CuSn SLID is chosen as the bonding technique due to its low cost, high hermeticity, and wafer-level compatibility [2]. CuSn SLID is a bonding technique in which Cu and Sn is deposited on the mating partners and heated to about 270 °C. At this temperature, the Sn melts and interdiffuses with the Cu, forming first the intermetallic (IMC) Cu6Sn5 and then Cu3Sn. After a time, all the Sn is consumed, and the final bond consists of Cu and Cu3Sn, both of which are highly hermetic and have a melting point far higher than that of Sn (Approximately 670 °C and 1000 °C for Cu3Sn and Cu respectively) [2].

**Fig. 1:** Cross-sectional model of packaged MBA with LWIR reflected light and areas for ARC highlighted with dashed lines (Not to scale).

Although silicon has a low absorption coefficient in the LWIR range [3], Fresnel reflections remain an issue. According to Fresnel's equations, ∼30% of the light will be reflected at a single Air-Si interface at normal incidences due to the large difference between the refractive indices of air and Si [4]. Since the light must traverse two such interfaces (see Fig. 1), some anti-reflective measures need to be taken at both interfaces. A common approach is to deposit an Anti-Reflective Coating (ARC) with typical reflectivity of <2% in the LWIR band. However, since a typical design requires 5–25 layers [5,6], all with potentially different coefficients of thermal expansion (CTE), these coatings are sensitive to changes in temperature.

An approach that has been shown to improve mechanical performance, is to dope an ARC consisting of multiple layers of TiO2/SiO2 with Zr-oxide [7]. These samples demonstrated improved hardness after annealing, but with limited increase in transmission (6%) and current demonstration limited to the white light region. Moth-eye structures, also referred to as anti-reflective gratings, is another technique that shows promise to reduce surface reflectivity, but is far less mature and requires more process steps than Anti-reflective coatings [5,8]. Moreover, there are concerns about the light scattering from moth-eye structures and its negative influence on image quality.

In this article, we have developed an ARC capable of retaining its anti-reflective properties and mechanical integrity up to 300 °C. This allows for the coating to be applied in situations where ARCs were previously thought unsuited, such as inside a package hermetically sealed by CuSn SLID, as shown in Fig. 1. This has been done by using a combination of a MgO adhesion layer, a simplified 2-layer structure, and a deposition temperature in-between room temperature and the bonding temperature.

The paper is organized as follows: We discuss the design of a six-layer ARC and two-layer ARC, the fabrication of the coatings on Si wafer, experimental measurements, and process optimizations. The results are then discussed before concluding the article.

### 1.1 Design

To perform this design, we have used a classical thin-film approach based on matrix formalism [9] to design and calculate a simple multilayer structure that would allow for the minimizing of the reflection coefficient in the 8–12 μm range for angles of incidence ranging from 0° to 30°. ZnS and YF_3_ were chosen as high and low refractive index materials respectively because they are classical infrared materials that both exhibit low absorption in the LWIR range. Two different structures were designed in the OptiLayer software using a needle approach [10]. First, a 6-layer anti-reflection was developed. Then, in order to limit the total stack thickness, the number of interfaces, and the bending caused by the stress and temperature dependence, the stack was eventually limited to a simpler 2-layer design with formula 1.04 H, 1.04 L where H represents a ZnS quarter wave layer and L a YF_3_ quarter wave layer, both at 10 μm. The refractive index at 10 μm wavelength of the ZnS and YF_3_ layers are equal to 2.257 and 1.363 respectively [11]. The thicknesses of the layers are equal to 1183 nm and 1935 nm respectively (see Table 1). This solution represents a compromise between minimizing the total thickness and minimizing the residual reflection of the final ARC.

**Table 1:** Composition of anti-reflective coatings.

Batch 1	Layer nr.	Material	Refr. Index	Thickness (nm)	Batch 2–4:	Material	Refr. Index	Thickness (nm)
	1	ZnS	2.257	1026		ZnS	2.257	1180
	2	YF_3_	1.363	1723		YF_3_	1.363	1908
	3	ZnS	2.257	151				
	4	YF_3_	1.363	969				
	5	ZnS	2.257	2102				
	6	YF_3_	1.363	1749				
Total				7719				3088

To verify the efficiency of the coatings, simulations were performed using the Optilayer software and the results for normal incidence and 30° incidence are presented in Fig. 2 below. We can see that the 2-layer coating theoretically reduces reflection to under 2% for a single air-Si interface, which is a great improvement compared to the original ∼30% of the bare Si wafer. Also, the 6-layer design has better overall performances than the 2-layer design, but sharper reflectance fluctuations at boundaries of the considered spectral region.

**Fig. 2:** Simulated results of the designed coatings at 0° and 30° angle of incidence.

### 1.2 Experimental fabrication

The ARCs were fabricated using a Bühler/Leybold Optics SYRUSpro 710 machine. ZnS layers were obtained from pure flakes placed in a Cu crucible while YF_3_ layers were obtained from pure granules that were preliminarily melted into a Mo liner. A focused electron beam (e-beam) was used to heat the material with a typical current of a few tens of mAmp for both materials. Specific e-beam patterns were developed in order to secure uniform evaporation of the material. 100 mm-diameter, 550 μm-thick silicon substrates were placed about 600 mm from the crucible on a rotating calotte to achieve layers with good uniformity over the substrate aperture. Thickness variation below 1% over the wafer aperture was achieved. Depositions were carried out at an initial pressure of about 10^−6^ mbar. Both materials were deposited at a rate of 0.3–0.5 nm/s. The deposition rates of the layers were controlled at a ±10% precision with a quartz crystal microbalance while the thickness was optically monitored with a Bühler OMS 5000. To achieve it, a white light beam is sent inside the chamber and the transmitted light is collected with an optical fiber which transmits it to a monochromator and a silicon detector. Due to the limited spectral range of the optical monitoring system, the layers were monitored at 870 nm wavelength, i.e. far from the operating wavelength of the antireflection coating meaning that the dispersion curve of the used materials must be well known over a broad spectral range. To verify that the thicknesses had been properly controlled, the transmission spectra were measured in the visible/near IR region using a PerkinElmer Lambda 1050 spectrophotometer after deposition, which showed very good agreement between theory and experiment.

The wafers with intact ARC were separated into multiple samples using a Disco 3220 Automated Dicing Saw. Heating of the samples was done in a Gravimetric Furnace LG, LAC.

The transmission of the structures is measured by a Nicolet is50 FTIR with a resolution of 4 cm^−1^ and 16 scans were performed for both the sample and the background measurements. The Nicolet is50 FTIR uses a Thermo Scientific Polaris™ source and a KBr-DLaTGS detector for the mid-to long-wave IR. The efficiency of the ARCs are measured by comparing a wafer with ARCs to an identical unprocessed wafer as presented in the results section. Measurements were made at 0° incidence and 30° incidence using a 3D-printed mount. Cross-sections of the coatings after dicing were taken by a Hitachi SU 3500 SEM.

The results of the FTIR measurements for a full wafer are also compared to simulations made in Zemax OpticStudio. These simulations were also performed by defining the material refractive indices vs wavelength (Si, Zns, YF3) assuming no absorption in the materials, and defining the ARC layer structure on one side and both sides of the Si wafer. The Polarization Ray tracing feature in Zemax allowed for the calculation of the optical transmission in the ARC-Si stack for the wavelength range measured.

### 1.3 Process optimization

The initial batch of ARC-coated wafers was composed of 6 layers (see Table 1). While this batch showed great promise to lower reflection as can be seen in the Optilayer simulations in Fig. 2, it disintegrated quickly after heating to 300 °C (see Fig. 3 a & b & Fig. 4 a & b). This is likely the result of the stress-induced in the layers by the CTE-mismatch between the Si wafer and the layers, which results in delamination [12]. These results lead to the 2-layer approach described below.

**Fig. 3:** ARC deposited at room temperature before (a) and after (b) subjected to 300 °C. Example of ARC delamination at room temperature as a result of deposition at 175 °C (c).

**Fig. 4:** SEM micrographs of a diced silicon wafer cross-section with a delaminated ARC (a) and the ARC that remained intact after heating (b). (For interpretation of the references to colour in this figure legend, the reader is referred to the Web version of this article.)

Few layers make the coating less susceptible to CTE-induced stress, but it is also known that ZnS has poor adhesion to Silicon. A 1–2 nm thick layer of MgO was therefore applied beneath ZnS for all designs and adhesion was confirmed by a scotch tape test.

Another important optimization turned out to be the choice of the deposition temperature of the ZnS and YF_3_ layers. It was found that if a too-low temperature is used during the deposition of the ZnS and YF_3_ layers, i.e. below 50 °C, delamination of the layers was observed when the sample was heated up to 300 °C (see Fig. 3 a & b & Fig. 4 a & b).

To overcome this challenge ZnS and YF_3_ were deposited at approximately 175 °C. This temperature was chosen as experience suggests that a higher temperature would cause deposition issues due to a too-large decrease in deposition rate, as suggested by Cox et al. [13]. This run resulted in a coating that cracked and delaminated when the samples were brought back to ambient temperature and pressure (see Fig. 3 c). The reason for this cracking is, in all likelihood, the same as that for the delamination seen in the first batch mentioned above.

Finally, an intermediate temperature of 100 °C was chosen for deposition. After deposition, this sample showed no cracking or delamination. The sample was then heated for 1 h at 300 °C, which did not affect the spectral properties or the mechanical stability of the coating (See Fig. 4).

## 2 Results

The transmission spectra of the wafers are presented in Fig. 5. For the wafers coated on one side, we see a 17% increase in transmission at 8 μm, with a steady decrease to about 10% at 12 μm (see Fig. 5 a). Below 8 μm there is still an overall increase in transmission, although quite uneven (see Fig. 5 b). Above 12 μm we see that the decrease in transmission improvement described continues. At 17.5 μm wavelength, the coated wafer crosses over to having increasingly lower transmission than an uncoated wafer as the coating was not designed for such a large spectral range. For the LWIR imaging, only the performance from 8 to 12 μm is relevant for the intended application. Measurements were made at 30° incidence as well. As can be seen from Fig. 5 c & d, these measurements also have a higher transmission at 8 μm wavelength which decreases as the wavelength increases. The difference between the normal incidence and 30° measurements is that the angled measurements show a slightly lower improvement, starting at 15%, and ending at 12% with an average of 14% increase in transmission.

**Fig. 5:** FTIR measurements comparing wafers with the final optimized ARC and without ARC in the intended wavelength range of 8–12 μm (a) and in the full measured 5–25 μm range (b). Same wafers measured with 30° incidence angle in the 8–12 μm range (c) and the 5–25 μm range (d). Comparison of an uncoated wafer, a single side coated, and a double side coated wafer (e). Simulated transmission comparison of an uncoated wafer, a single side coated, and a double side coated wafer from Zemax Opticstudio (f).

At 15 μm wavelength, some dips and spikes can be seen. These arise because CO_2_ has an absorption peak at 14.9 μm wavelength [14]. This means that when the chamber of the FTIR is opened and closed by the operator, to go from background measurement to measurement of the sample, slight variations in the CO_2_ concentration will cause a dip, or a spike, as seen in the aforementioned figures.

SEM images of the final coating revealed no delamination after heating, meaning the ARC also maintained good adhesion and mechanical integrity (see Fig. 4).

As an additional test, a wafer had both sides covered with the successful ARC. These wafers were also run through heat cycling and measured in the FTIR. The results in Fig. 5 e show that coating the wafer on both sides provides an additional 15% increase in transmission. It is clear that in the 8–12 μm range, the difference between an uncoated and single-side coated wafer, is very similar to the difference between a single-side and a double-side coated wafer.

Simulated transmission results for a full wafer is also presented in Fig. 5 f. Ignoring the dip in transmission at 9 μm wavelength, which may be explained by the high presence of oxygen in Czochralski silicon [15], results show a very good correlation. The simulations show slightly higher transmission than the experiments, most likely due to the scattering experienced in the FTIR measurements.

## 3 Discussion

A detailed process description for an effective heat-resistant ARC coating has been presented, along with three unsuccessful ones.

At first, we tested the design and more specifically the number of layers. It turned out that we opted for the simplest design even if it resulted in lower optical performances. This choice is linked to the fact that the thickness of the 2-layer design is less than half of that of the 6-layer coating. Since the temperature-induced deformation is linked to the total stack thickness [16], this assists in minimizing it. In addition, minimizing the number of layers minimizes the number of interfaces. This further reduces the chances of delamination for the 2-layer design.

Another important optimization was the choice of the deposition temperature of the ZnS and YF_3_ layers. We demonstrated that depositing the layers at a too high or too low temperature does not result in an antireflection coating that is stable at both 25 °C and 300 °C. To better understand this process, one needs to keep in mind that stress has three contributions [17]:

(1) $$\sigma_{tot}=\sigma_{\mathrm{int}}+\sigma_{therm}+\sigma_{env}$$

where σ_tot_, σ_int_, σ_therm_, and σ_env_ is total stress, intrinsic stress, thermal stress, and environmental stress respectively. Intrinsic stress is linked to the factors such as material and the deposition procedure, while the thermal stress depends on the deposition and usage temperatures, and environmental stress can be affected by, for example, water adsorption. In this project, the most problematic stress being the thermal stress, it is clear that depositing coatings at a low temperature allows minimization of stress at low temperature, but maximizes it when the temperature is increased to 300 °C afterward. Increasing the deposition temperature too much, however, minimizes the stress at 300 °C, but, in this case, leads to cracking at low temperatures when cooling down, as seen in Fig. 3 b. It is also interesting to note that the damage is different for the two types of samples. A coating deposited a room temperature and then annealed at 300 °C shows complete destruction of the sample (flaking). The sample coated at 175 °C, on the other hand, is delaminated when brought back to room temperature. These two visual effects reveal that the origins of delamination (i.e. the relative stresses) are probably different for the two studied cases. However, since these two samples do not match the project requirement, no further analysis was performed.

To overcome these issues, we found that using an intermediate temperature of 100 °C, right in between the two previous temperatures, allows for minimizing of the thermal stresses, and therefore the overall stress at both room temperature and 300 °C (See Fig. 4).

The successful ARC was compared to a blank wafer using an FTIR spectrometer in transmission mode. It should be noted that the FTIR spectrometer measurements include losses due to scattering, reflection from the uncoated side of the wafer, and absorption in the silicon and coating. These factors explain the difference between the results seen in the thin-film simulations and the experimental results. In a final packaged device, thinner silicon with lower absorption may be used, and both sides of the silicon cap will be coated, resulting in higher transmission than presented here. Moreover, high resistivity Si wafer can be used which has lower intrinsic absorption as compared to the wafers used in this study, especially at 9 μm wavelength [15].

The coating developed in this study demonstrate lower transmission than coatings with no heat-resistance requirement, such as the 4-layer Si3N4/SiO2 coating developed by Zeng et al. [18]. This is unsurprising considering our simulations of our own 6-layer coating also demonstrated higher transmission than the final two-layered heat-resilient one. Our coatings also demonstrate lower transmission than some of the moth-eye structures presented in the literature [5]. As mentioned in the introduction, however, these structures require more process steps and raise concerns about scattering for thermal imaging applications. For a heat-resilient ARC that is easily integrated in an existing process flow, the transmission results demonstrated are very promising, as can be seen by comparison with the 6% increase in transmission demonstrated by the mechanically robust and heat-resilitent coating developed by Zambrano-Mera et al. [7].

While a wafer with coating on both sides is demonstrated, only one side will need heat-resistant coating in the final product. This is because the coating on the outside of the final Si lid can be done as the final step of the packaging process, which means it will not have the same stringent requirements when it comes to temperature resistance. This means more traditional coating with more layers and higher transmission may be selected and deposited at room temperature on the outside of the cap wafer [19].

Another consideration is that we have deposited the coatings on flat wafers. If the coating is to be used as shown in Fig. 1 the coating will need to be deposited in a cavity, on a micromachined surface. Fortunately, the deposition method used, i.e. e-beam sputtering, is compatible with using a shadow mask, as long as the mask material has a CTE similar to silicon [20]. Simulations have also shown that the roughness in the cavity as a result of micromachining, i.e. wet- or direct ion etching, will not negatively impact the transmission [21].

## 4 Conclusion

In this article, a detailed process description and development of an AR coating able to maintain its anti-reflective properties up to 300 °C for 1 h have been presented. This is beyond the requirements for a CuSn SLID bonding process, which is usually done at about 270 °C for 30 min [22]. In the targeted LWIR range of 8–12 μm, the ARC demonstrated an average improvement of more than 15% for normal incidence and 13% for 30° incidence when compared to an uncoated wafer. This was achieved by using only two layers (ZnS and YF_3_), a thin MgO adhesion layer, and deposition at 100 °C. Three unsuccessful attempts for making such a coating have also been presented. These coatings consisted of more layers and were deposited at room temperature or 175 °C, which caused them to delaminate upon temperature cycling to 300 °C.

This coating may be directly employed in MBA-based thermal cameras, but the techniques and considerations made here also have potential applications where a thermal camera must go through high temperatures before or during operation, such as in space and subsea.

## Data availability statement

Data will be made available on request.

## Credit author statement

Phillip Papatzacos: Investigation, Methodology, Validation, Writing – Original Draft, Visualization, tests and analysis of the film **M. Nadeem Akram:** Conceptualization, Methodology Writing – Review & Editing, Supervision **Julien Lumeau:** Conceptualization, Methodology Writing – Review & Editing, Supervision **Olivier Hector:** Fabrication, tests and analysis of the film **Frédéric Lemarquis:** Design of the film, Methodology Writing – Review & Editing **Antonin Moreau:** Fabrication, Test and analysis of the film **Per Ohlckers:** Funding acquisition, Project administration, Supervision.

## Declaration of competing interest

The authors declare that they have no known competing financial interests or personal relationships that could have appeared to influence the work reported in this paper.
